The article "Analyzing the Relationship among Social Capital, Dynamic Capability, and Farmers' Cooperative Performance Using Lightweight Deep Learning Model: A Case Study of Liaoning Province" was retracted in 2023. Reasons: signs of a paper mill; suspected computer-generated content; unreliable results or conclusions; concerns about the data.

# Analyzing the Relationship among Social Capital, Dynamic Capability, and Farmers' Cooperative Performance Using Lightweight Deep Learning Model: A Case Study of Liaoning Province

**DOI:** 10.1155/2023/7064236

**Published:** 2023-03-01

**Authors:** Simeng Zhang, Dongli Wu

**Affiliations:** School of Economics and Management, Shenyang Agricultural University, Shenyang 110000, China

## Abstract

The purpose of this study is to understand the relationship between social capital and the performance of Farmers' Cooperatives (Cooperatives) and explore the internal mechanism of social capital affecting the performance of Cooperatives. This work selects two dimensions: cognitive social capital (CSC) and structural social capital (SSC), as indexes to measure the social capital of Cooperatives. An analytical framework is proposed: “Social capital-Dynamic capabilities-Organizational performance.” First, according to the characteristics of Cooperatives, it determines the most appropriate index values and preprocesses the original data. Statistical Product and Service Solutions (SPSS) and Analysis of Moment Structure (AMOS) 25.0 software are used for factor analysis. A financial performance evaluation model of Cooperatives based on backpropagation neural network (BPNN) is constructed. Then, based on the survey data of 212 Cooperatives in Liaoning Province, the structural equation model (SEM) is used to test the interaction path between “Social capital-Dynamic capacity-Organizational performance.” The results show that SSC's standardized regression coefficients (SRCs) on Cooperatives' economic benefits and member satisfaction are 0.208 and 0.095, respectively, significant at 1%. The actual case analysis concludes that the larger the scale of the structural network embedded in Cooperatives is, the more conducive it is to obtaining extensive resources. As such, Cooperatives can absorb the advanced experience and compensate for the weakness of lack of internal resources and experience. The SRC of CSC on Cooperatives' economic benefits is 0.336, and the *P* value is 0.204, indicating an insignificant impact of CSC on Cooperatives' economic benefits. This work considers environmental variability, uses dynamic capacity as an independent variable, opens the “black box” between social capital and the performance of Cooperatives, and reveals the intermediate path between the two.

## 1. Introduction

Farmers' Cooperatives (hereafter Cooperatives) are the core carrier of small-scale farmers' organizations and play an essential role in increasing farmers' income and achieving common prosperity. They are defined as an organization based on rural household contract management. They aim to realize mutual assistance among their members by providing services, such as sales, processing, transportation, and storage of agricultural products and technology. They also offer information related to agricultural production and management. Professional Cooperatives are organizations similar to companies and have unity in finance and decision making. They have a certain organizational structure, and their members enjoy certain rights and responsibilities. With the promulgation of the Cooperative Law, the number of Cooperatives in China has increased rapidly. By April 2021, registered Cooperatives following the law have reached 2,259,000, and Cooperative members have accounted for more than 50% of the total number of farmers in China [1]. The recent documents also pointed out that developing new agricultural economies, such as Cooperatives, small farmers, and family farms, has rapidly promoted rural economic growth. The No. 1 Central Document issued in 2021 stated, “We should focus on Cooperatives and family-run farms and encourage the development of various forms of medium-sized enterprises.” As the core of organizational behavior, performance evaluation can help enterprises explore their problems [2–4].

The article "Analyzing the Relationship among Social Capital, Dynamic Capability, and Farmers' Cooperative Performance Using Lightweight Deep Learning Model: A Case Study of Liaoning Province" was retracted in 2023. Reasons: signs of a paper mill; suspected computer-generated content; unreliable results or conclusions; concerns about the data.

The lightweight deep learning (DL) model simplifies network computing and accelerates network operation. It uses the Relu function and structural optimization to reduce the number of channels and increase network layers to accelerate the network. It was first applied to prediction problems. However, with the continuous deepening of research, many scholars have applied it to evaluation problems. Luo and Ren (2021) established an enterprise performance evaluation model based on neural network (NN) and optimized the model using factor analysis and a genetic algorithm (GA). The main factors affecting enterprise performance were analyzed. Then, it quantitatively analyzed the performance of the acquirer in the merger and acquisition (M&A) commitment period under the income compensation mechanism. The corresponding assumptions and evaluation indicators were established [5]. Liang and Li [6] proposed a spatial network-distributed data mining algorithm based on backpropagation NN (BPNN) to evaluate personnel performance effectively. Multi-input and multi-output (MIMO) spatial network data were built in the cloud computing environment to analyze the data structure. Massive amounts of data were compressed through time-frequency feature extraction (TFFE). The data features were matched combined with an adaptive matched filtering method. To improve the data mining accuracy, BPNN was used to classify and recognize the extracted data features to optimize data mining [6]. He and Zhang [7] studied the phosphorus content prediction model based on principal component analysis (PCA) and BPNN. The research reduced the index dimension affecting the end-point phosphorus content and eliminated the correlation between the indexes. The experimental results showed that the prediction accuracy of the designed model was the highest, and PCA improved the model's generalization ability. The actual production results showed that the designed model could predict the end-point phosphorus content [7]. It can be found from the current research that DL technology has been used in scientific research. However, the model output needs to be further optimized.

The article "Analyzing the Relationship among Social Capital, Dynamic Capability, and Farmers' Cooperative Performance Using Lightweight Deep Learning Model: A Case Study of Liaoning Province" was retracted in 2023. Reasons: signs of a paper mill; suspected computer-generated content; unreliable results or conclusions; concerns about the data.

This work selects cognitive social capital (CSC) and structural social capital (SSC) indexes to measure the Cooperatives' social capital and constructs an analytical framework: “Social capital-Dynamic capabilities-Organizational performance.” First, according to the characteristics of Cooperatives, it determines the most appropriate index value and preprocesses the original data. Statistical Product and Service Solutions (SPSS) is used for factor analysis, and Cooperatives' BPNN financial performance evaluation model is constructed. Then, based on the survey data of 212 Cooperatives in Liaoning Province, this work uses structural equation model (SEM) to test the interaction path between “Social capital-Dynamic capability-Organizational performance.” The research innovation is to apply DL technology to solving agricultural problems and explore the new social development path.

## 2. Model Implementation and Research Hypothesis

### 2.1. BPNN Construction

BPNN comprises the input, output, and hidden layers and is implemented based on the BP algorithm. The specific implementation steps are as follows. First, it inputs the data into the network structure and outputs the results after three levels of processing. The forward propagation process ensures the independency of interlayer nodes, and different levels can only affect the forward or backward section nodes. The BP mechanism will be excited when the expected error and output result exceed the acceptable range. The error signal will return in reverse according to the propagation direction. The error between the expected value and output result will be ideal by continuously determining the neuron connection weight [8].

#### 2.1.1. Number of Network Layers

A typical BPNN includes one input layer, one or more hidden layers, and one output layer. The number of hidden layers must be determined before model implementation. Generally, a single hidden layer NN will be preferred in actual problems. Nevertheless, the mapping accuracy often improves as the number of hidden layers increases despite the resultant complex structure. Meanwhile, increased hidden layers mean a multiplication of the training and learning cycle, sometimes leading to overfitting. Given the above analysis, this work establishes a BPNN structure with one hidden layer to evaluate the performance of Cooperatives [9–11].

The article "Analyzing the Relationship among Social Capital, Dynamic Capability, and Farmers' Cooperative Performance Using Lightweight Deep Learning Model: A Case Study of Liaoning Province" was retracted in 2023. Reasons: signs of a paper mill; suspected computer-generated content; unreliable results or conclusions; concerns about the data.

#### 2.1.2. Determination of Node Number

The performance evaluation indicator corresponds to the number of nodes in the BPNN input layer. This section selects 13 performance evaluation indicators (PEIs) to evaluate the efficiency of Cooperatives, as detailed in Figure 1.

The dependent variable corresponds to the output layer node of the BPNN, and the specific quantity setting needs to be based on the actual scenarios. This work chooses the performance of Cooperatives as the dependent variable, which contains only one variable. Accordingly, the BPNN's output layer node number is set to one.

So far, no unified method has been used to determine the number of hidden layer nodes. Too few hidden layer nodes will have a certain impact on the fitting effect. In contrast, too many nodes will lead to prolonged learning time, resulting in overfitting [12, 13]. Fortunately, there are methods to determine the range of hidden layer nodes, as

(1) $$\begin{array}{c} K=\sqrt{m+n}+d. \end{array}$$

In (1), *m*, *n*, and *K* are the number of nodes in the input, output, and hidden layers, respectively. *d* is a random number ∈ [1, 10]. The input layer contains 13 nodes, and the output layer has one node. According to (1), the number of hidden layer nodes can be calculated as five to 13. Then, through multiple experiments, the ideal model effect can be obtained when the number of hidden layer nodes is 10.  Figure 2 unfolds the constructed BPNN structure.

### 2.2. Influencing Factors of Cooperatives' Performance

#### 2.2.1. Social Capital on the Performance of Cooperatives

Structural social capital (SSC) is a social relationship network formed by Cooperatives and external subjects. The larger the scale of the social network is, the more information and resources the Cooperative contains in the embedded network. Extensive social relations can help Cooperatives obtain financial capital, key technologies, and management experience. As such, Cooperatives can maintain information and knowledge advantages and promote economic benefits. The personalized relationship established by frequent social interaction accelerates the flow of intangible resources with high value and enables Cooperatives to obtain more high-quality information and resources, which is also beneficial to Cooperatives' economic benefits [14].

The article "Analyzing the Relationship among Social Capital, Dynamic Capability, and Farmers' Cooperative Performance Using Lightweight Deep Learning Model: A Case Study of Liaoning Province" was retracted in 2023. Reasons: signs of a paper mill; suspected computer-generated content; unreliable results or conclusions; concerns about the data.

In addition, through close contact with scientific research institutions and government agencies, Cooperatives can provide members with more technology and information, thereby improving member satisfaction. Cognitive social capital (CSC) is the degree of trust between members within a Cooperative, between members and managers, and the degree of recognizing values. Trust and common values are the basis for stable cooperation among members. A stable organizational relationship is conducive to preventing opportunistic behavior and reducing the internal transaction costs of Cooperatives. Transaction cost reduction frees up the flow of information and funds within Cooperatives, bringing higher economic benefits.

Therefore, CSC plays a positive role in improving the economic benefits of Cooperatives. On the other hand, trust and common values can promote communication among Cooperative members and action coordination among members. In a collective action, the needs for social communication and the emotion of members are met by strengthening the emotional communication between members. The perceived evaluation of members can be improved [15]. In view of this, hypothesis 1 is proposed:

  H1: Social capital has a positive impact on the performance of Cooperatives
  H1a: SSC has a positive impact on the economic benefits of Cooperatives
  H1b: CSC has a positive impact on the economic benefits of Cooperatives
  H1c: SSC has a positive impact on the satisfaction of Farmers' Cooperative members
  H1d: CSC has a positive impact on the satisfaction of Farmers' Cooperative members

#### 2.2.2. Social Capital on the Dynamic Capability of Cooperatives

Resources are the basis of capabilities. Dynamic capabilities must be built on valuable, scarce, inimitable, and irreplaceable resources. Social capital expands and strengthens the connection between Cooperatives and external organizations with unique resources, providing resource reserves for Cooperatives. This shows that social capital has an important impact on the formation of the dynamic capacity of Cooperatives. Specifically, a single connection between a Cooperative and an external subject will be difficult to cope within a dynamic environment. The diversity and scope of interorganizational relations are the main sources of dynamic capabilities. SSC broadens the scope of external exchanges and contacts of cooperatives, enabling them to obtain a wide range of information. As such, Cooperatives can perceive the changes in the external environment timely and identify opportunities and threats in the market in this process.

At the same time, close social ties promote Cooperatives to learn and absorb advanced management experience and operation processes more effectively. The ties help Cooperatives improve organizational practices and operational efficiency [16, 17]. CSC improves the relationship quality among members and between members and managers. High relationship quality represents a transparent and open cooperative relationship, improving members' willingness to share information with cooperatives. Accelerating the flow of intangible resources enables Cooperatives to obtain better information, comprehensively understand the market environment, and thus have a more agile understanding of environmental changes. In addition, recognizing organizational values strengthens the common language between members and Cooperatives. It promotes deeper interaction and communication, helps Cooperatives find deficiencies in operation in time, and improves operational efficiency through the organizational change in a shorter time. In view of this, hypothesis 2 is proposed:

  H2: Social capital has a positive impact on the dynamic capability of Cooperatives
  H2a: SSC has a positive impact on the environmental perception of Farmers' Cooperatives
  H2b: CSC has a positive impact on Cooperatives' environmental perception
    H2c: SCC has a positive impact on the organizational changeability of Cooperatives
  H2d: CSS has a positive impact on the organizational changeability of Cooperatives

The article "Analyzing the Relationship among Social Capital, Dynamic Capability, and Farmers' Cooperative Performance Using Lightweight Deep Learning Model: A Case Study of Liaoning Province" was retracted in 2023. Reasons: signs of a paper mill; suspected computer-generated content; unreliable results or conclusions; concerns about the data.

#### 2.2.3. Dynamic Capability on the Performance of Cooperatives

Against a dynamic, complex, and competitive external environment, whether Cooperatives can maintain their competitive advantage and remain invincible depends on their adaptability to the external environment. Under the defensive stress mechanism, Cooperatives have the organizational ability to adapt to and respond to changes in the external environment [18]. Environmental perception ability is the primary factor of dynamic capability, and its core is information, which is the micro basis for the impact of dynamic capability on organizational performance. By scanning and perceiving relevant government policies, industrial structure, and consumer demand, Cooperatives can quickly identify market opportunities in the environment, create first-mover advantages, and boost economic benefits. Cooperatives can seize new market opportunities and enhance their voice by developing new products and applying new technologies.

With the increasingly dominant position in the market, Cooperatives can strive for more rights and interests for members to have a sense of organizational identity. Organizational changeability is evolutionary adaptability to eliminate the adverse effects of organizational inertia and path dependence. It helps organizations obtain a lasting competitive advantage. By changing the basic constituent units, such as resources and processes, and then restoring the matching with the external environment, Cooperatives can improve operational efficiency. Then, they can respond quickly to the fierce competition, regain competitiveness, and improve economic benefits. In addition, the ability of organizational change will drive Cooperatives to adjust redundant resources and management concepts. Further, it improves the application mode of Cooperatives, promoting Cooperatives to accelerate product innovation and improve service quality. Thereby, it improves members' recognition and satisfaction with Cooperatives [19–21]. In view of this, hypothesis 3 is proposed:

  H3: Dynamic capability has a positive impact on the performance of Cooperatives
  H3a: Environmental perception has a positive impact on the economic benefits of Cooperatives
  H3b: The ability of organizational change has a positive impact on the economic benefits of Cooperatives
  H3c: Environmental perception has a positive impact on the satisfaction of Farmers' Cooperative members
  H3d: The ability of organizational change positively impacts the satisfaction of Farmers' Cooperative members

The article "Analyzing the Relationship among Social Capital, Dynamic Capability, and Farmers' Cooperative Performance Using Lightweight Deep Learning Model: A Case Study of Liaoning Province" was retracted in 2023. Reasons: signs of a paper mill; suspected computer-generated content; unreliable results or conclusions; concerns about the data.

#### 2.2.4. Moderating Role of Dynamic Capability

Existing studies have confirmed that the relationship between social capital and organizational performance is a complex and dynamic process. The new knowledge and information obtained by Cooperatives embedded in social networks are difficult to promote organizational performance directly. They often gradually maximize the resource value by constantly absorbing and utilizing new knowledge [22, 23]. The larger the scale of the Cooperative's external relationship network is, the more market information it can obtain, helping to capture emerging market opportunities. Thus, Cooperatives can respond to market demand and changes timely and turn potential opportunities into competitive advantages. The more favorable the position of the Cooperative in the external relationship network is, the more heterogeneous resources it can obtain. This helps the Cooperative integrate internal and external resources and allocate resources according to the external environment changes.

Innovating products to meet the market's diversified needs can improve Cooperatives' performance. The more Cooperative and other relational network subjects have a common language, the more they can reduce ambiguity and misunderstanding and promote the tacit knowledge exchange between them. This helps give play to the synergy of network members to achieve knowledge sharing and resource complementarity. In short, dynamic capabilities play an important role as a bridge between social capital and the performance of Cooperatives [24, 25]. In view of this, hypothesis 4 is proposed:

  H4: Dynamic capability plays a moderating role between social capital and the performance of Cooperatives.

The article "Analyzing the Relationship among Social Capital, Dynamic Capability, and Farmers' Cooperative Performance Using Lightweight Deep Learning Model: A Case Study of Liaoning Province" was retracted in 2023. Reasons: signs of a paper mill; suspected computer-generated content; unreliable results or conclusions; concerns about the data.

The proposed hypothetical model is illustrated in Figure 3.

### 2.3. Questionnaire Survey (QS) Design

#### 2.3.1. Explanatory Variable

Social capital is the collection of resources embedded in Cooperatives' social relationship network. This section divides Cooperatives' social capital into two dimensions: structural and cognitive. The five-point Likert scale assigns and scores the indexes [26, 27]. SPSS and Analysis of Moment Structure (AMOS) 25.0 software are used for factor analysis. The specific item design is shown in Figure 4.

#### 2.3.2. Mediating Variable

Based on the original scale, combined with the organizational characteristics and operation of Cooperatives, a dynamic capability scale for measuring such organizational forms as Cooperatives is constructed. The SPSS and the AMOS 25.0 software are used for factor analysis. The specific dynamic capability scale is shown in Figure 5.

## 3. Performance Evaluation and Empirical Analysis

The empirical data come from the special survey of 212 Cooperatives in Liaoning Province conducted by the school of Economics and Management of Shenyang Agricultural University from January to September 2021. The subjects are Cooperatives running for three years or more and have been officially registered with the Department of Industry and Commerce.

### 3.1. Performance Evaluation

Next, the proposed BPNN-based Cooperatives-oriented performance evaluation model is verified through simulation experiments on randomly selected 30 groups of Farmers' Cooperative data.  Figure 6 describes the output results.

As in Figure 6(a), the expected output of Cooperatives in 2021 is consistent with the actual output. The average and maximum relative errors are 0.0036 and 0.025, respectively. The mean square error (MSE) is 0.00000095, far less than the preset value of 10^−5^. The prediction results meet the requirements of the simulation test.

Subsequently, the performance score of Cooperatives from 2019 to 2021 is calculated through the proposed BPNN-based Cooperatives-oriented performance evaluation model. Then, the influencing factors of Farmers' Cooperative performance are analyzed according to the specific score results and the proposed hypothetical model.

First, according to the established PEIs of Cooperatives, data of the 13 indicators of Cooperatives in Liaoning Province from 2019 to 2021 are collected and calculated. The specific data are plotted in Figure 7.

The article "Analyzing the Relationship among Social Capital, Dynamic Capability, and Farmers' Cooperative Performance Using Lightweight Deep Learning Model: A Case Study of Liaoning Province" was retracted in 2023. Reasons: signs of a paper mill; suspected computer-generated content; unreliable results or conclusions; concerns about the data.

Here, the 13 indicator data in Figure 7 are input into the proposed BPNN-based Cooperatives-oriented performance model, the performance evaluation model. Accordingly, the performance score of Liaoning Cooperatives from 2019 to 2021 is estimated and displayed in Figure 8.

According to Figure 8, the performance scores of Cooperatives in Liaoning Province from 2019 to 2021 are all negative, and the actual operation condition is poor. The performance level has declined rapidly after a small increase in the past three years. The performance score of Cooperatives in the recent three years gives an early warning to their backward and unscientific operation and management. The results reflect some problems in Cooperatives' strategic decision-making development and daily business. Thus, it is urgent to explore the causes and eliminate relevant problems through in-depth analysis.

### 3.2. Results of Influencing Factors of Farmers' Cooperative Performance

In this survey, 15–25 Cooperatives are selected from the list of Cooperatives in each prefecture and city, and QSs are distributed. Overall, 250 QSs are distributed, and 182recovered, with 144 valid. The characteristics of sample data are reflected in Figure 9.

Then, SPSS 25.0 tests the construct validity, discriminant validity, and combination reliability. The results are charted in Figure 10.

Figure 10 implies that the Cronbach's *α* of each latent variable is between 0.761 and 0.871, higher than the minimum requirement of 0.60. Thus, each scale and its items have passed the reliability test. Further, the factor load of each latent variable measurement item is higher than 0.60, and the AVE is greater than the standard evaluation value of 0.50. Thus, all scales and their items have good constructive validity.

The main variables are latent variables that are difficult to observe directly. This section uses SEM to study social capital, dynamic capability, and the performance of Cooperatives. It tests the model's relationship and interaction between explicit, latent, and error variables. AMOS 25.0 is used to verify the fitting degree of the hypothetical model. The results show that the overall model has good adaptability, and the fitting is ideal. *e*1–*e*26 represent different influence factors. The analysis results of the overall model are shown in Figure 11.

Figure 11 shows that SSC's standardized regression coefficients (SRCs) on Cooperatives' economic benefits and member satisfaction are 0.208 and 0.095, respectively, significant at 1%. Thus, the larger the scale of the structural network embedded in Cooperatives, the more conducive it is to obtain a wide range of resources, absorb the advanced experience, and make up for the weakness of lack of internal resources and experience. The results are reflected in Cooperatives' performance level. Hypotheses H1a and H1c are verified. The SRC of CSC on Cooperatives' economic benefits is 0.336, and the *P* value is 0.204. Hence, the impact of CSC on Cooperatives' economic benefits is insignificant, and hypothesis H1c is invalid.

The article "Analyzing the Relationship among Social Capital, Dynamic Capability, and Farmers' Cooperative Performance Using Lightweight Deep Learning Model: A Case Study of Liaoning Province" was retracted in 2023. Reasons: signs of a paper mill; suspected computer-generated content; unreliable results or conclusions; concerns about the data.

The possible reasons are, on the one hand, the members' own economic strength and knowledge level are limited. Even if they trust the organization, it is difficult to provide scarce resources for Cooperatives to help members accumulate capital and develop markets. On the other hand, members' trust in the organization can alleviate the dilemma of collective action and is conducive to the long-term development of Cooperatives. However, the impact on economic benefits is usually lagging. This work uses cross-sectional data to analyze the impact of CSC on the level of economic benefits in the current period, so H1c is not established. The SRC of CSC on the Cooperative members' satisfaction is 0.136, significant at 1%. Hypothesis H1d is verified.

The SRCs of SSC and CSC on the environmental perception of Cooperatives are 0.169 and 0.157, respectively, significant at the level of 1%. Hypotheses H2a and H2b are verified. The standardized coefficients of SSC and CSC on the organizational changeability of Cooperatives are 0.332 and 0.214, reaching a significant level. Hypotheses H2c and H2d are also verified. Specifically, SCC provides an opportunity for Cooperatives to learn advanced management experience, promotes Cooperatives to examine their shortcomings, and then triggers organizational change. CSC accelerates the exchange of tacit knowledge within Cooperatives and promotes them to design new products and technologies under the action of trust.

The SRCs between environmental perception ability, organizational changeability, and economic benefits of Cooperatives are 0.243 and 0.351, respectively. The path coefficients reach a significant level. Thus, hypotheses H3a and H3b are verified. Specifically, environmental perception can help Cooperatives gain the market initiative to promote them to seize market opportunities and obtain more economic benefits. By eliminating organizational inertia and path dependence, organizational changeability enables Cooperatives to respond strategically to the external environment, exerting their competitive advantages and obtaining higher income.

The SRCs between environmental perception ability, organizational changeability, and member satisfaction are 0.142 and 0.227, respectively, significant at 1% and 5%. Hence, hypotheses H3c and H3d are verified. Of these, environmental perception ability makes Cooperatives pay more attention to innovation. It continuously consolidates Cooperatives' industry status through product research and development and gives members a sense of organizational identity. As a result, member satisfaction is improved. The ability of organizational change promotes the adoption of updated technology and the improvement of the management system of Cooperatives, meets the service needs of members, and enhances the satisfaction of members.

The article "Analyzing the Relationship among Social Capital, Dynamic Capability, and Farmers' Cooperative Performance Using Lightweight Deep Learning Model: A Case Study of Liaoning Province" was retracted in 2023. Reasons: signs of a paper mill; suspected computer-generated content; unreliable results or conclusions; concerns about the data.

The path analysis in SEM is listed in Table 1.

According to Table 1, the total effect of social capital on Farmers' Cooperative performance is 0.897. The direct effect is 0.439, partly from the direct effect of SSC on the economic benefits and member satisfaction of Cooperatives and partly from the direct effect of CSC on the satisfaction of Farmers' Cooperative members. The indirect effect is 0.458, which comes from four indirect paths. Specifically, the intermediary path of SSC ⟶ organizational changeability ⟶ economic benefits has the greatest intensity, 0.117, accounting for 13.04% of the total effect. CSC cannot directly affect the economic benefits of Cooperatives but can indirectly promote the improvement of benefits through dynamic capability. Thus, dynamic capability plays a partial moderating role in the impact of social capital on the performance of Cooperatives.

Further, this section uses the Bootstrap method to verify the moderating role of dynamic capabilities. This method regards the existing sample space as the whole of the research object and carries out repeated sampling with a return in the sample space. AMOS 25.0 extracts 2,000 times at 95% confidence level. Percentile and bias-corrected methods are used to test the effect value of mediation. If the confidence interval obtained from the indirect effect result does not contain 0, there is a moderating effect. The results obtained are shown in Table 2. Among the multiple intermediate paths from social capital to Cooperative performance, the high and low ranges of indirect effects do not contain 0. Therefore, there is a moderating effect between social capital and Cooperative performance, and hypothesis H4 holds.

## 4. Conclusion

Cooperatives positively affect farmers' income and the common prosperity goal and are the main form of the small-scale farmers' organization. In order to understand the relationship between social capital and the Cooperatives' performance, this work constructs a lightweight DL model to calculate and analyze the financial performance scores of Cooperatives in Liaoning Province from 2019 to 2021. Then, it selects CSC and SCC indexes to measure the Cooperatives' social capital and constructs an analytical framework of “Social Capital-Dynamic capability-Organizational performance.” Based on the survey data of 212 Cooperatives in Liaoning Province, it uses the SEM to test the interaction path between the three. The research results have proved the hypotheses, indicating that the research is reasonable, and the obtained model can also be applied to the actual production process.

The article "Analyzing the Relationship among Social Capital, Dynamic Capability, and Farmers' Cooperative Performance Using Lightweight Deep Learning Model: A Case Study of Liaoning Province" was retracted in 2023. Reasons: signs of a paper mill; suspected computer-generated content; unreliable results or conclusions; concerns about the data.

This work explores the internal mechanism of social capital affecting Cooperatives' performance, but there are still some limitations. First, the sample data are cross-sectional, collected simultaneously rather than longitudinal research, without considering the possible time effect between the main variables. Subsequent research can use time series data to deepen the research. Second, this work only samples Cooperatives in Liaoning Province and cannot reflect the development status of Cooperatives in different regions. In the future, it is expected to expand the sample range and do more extensive empirical research to enhance the universality of the conclusions.

## Figures and Tables

**Figure 1:** Operational PEIs of Cooperatives.

**Figure 2:** BPNN structure.

**Figure 3:** Hypothetical model.

**Figure 4:** Measurement of explanatory variables.

**Figure 5:** Measurement of mediating variables.

**Figure 6:** Network output results. (a) Error between actual output and expected output. (b) Inspection error and error percentage.

**Figure 7:** Index data of Cooperatives.

**Figure 8:** Performance score.

**Figure 9:** Basic information of survey samples. (a) Product category. (b) Education level of the chairman. (c) Member size. (d) Asset size.

**Figure 10:** Results of reliability and validity analysis of the scale (CR: composite reliability; AVE: average variance extraction).

**Figure 11:** SEM and path calculation results. Note. ^*∗*^, ^*∗∗*^, and ^*∗∗∗*^ are significant at the level of 10%, 5%, and 1%, respectively, and dotted lines represent the insignificant regression paths.

**Table 1:** Model path coefficient and standardization effect.

Model path	Overall effect	Direct effect	Indirect effect
SSC ⟶ economic benefits	0.795	0.208	0.323
CSC ⟶ economic benefits	0.113	0.000	0.113
SSC ⟶ member satisfaction	0.573	0.095	0.278
CSC ⟶ member satisfaction	0.349	0.136	0.113
SSC ⟶ environmental perception	0.350	0.169	0.000
CSC ⟶ environmental perception	0.157	0.157	0.000
SSC ⟶ organizational change ability	0.571	0.332	0.000
CSC ⟶ organizational change ability	0.214	0.214	0.000
Environmental perception ⟶ economic benefits	0.243	0.243	0.000
Organizational change ability ⟶ economic benefits	0.351	0.351	0.000
Environmental perception ⟶ member satisfaction	0.342	0.142	0.000
Organizational change ability ⟶ member satisfaction	0.277	0.227	0.000
Social capital ⟶ farmers' cooperative performance	0.897	0.439	0.458
Dynamic capability ⟶ economic benefit	0.594	0.594	0.000
Dynamic capability ⟶ member satisfaction	0.369	0.369	0.000

The article "Analyzing the Relationship among Social Capital, Dynamic Capability, and Farmers' Cooperative Performance Using Lightweight Deep Learning Model: A Case Study of Liaoning Province" was retracted in 2023. Reasons: signs of a paper mill; suspected computer-generated content; unreliable results or conclusions; concerns about the data.

**Table 2:** Moderating effect test.

Model path	Bias-corrected		Percentile method	
	Lower	Upper	Lower	Upper
SSC ⟶ environmental perception ⟶ economic benefits	0.113	0.268	0.113	0.267
SSC ⟶ organizational change ability ⟶ economic benefits	0.027	0.458	0.026	0.459
SCC ⟶ environmental perception ⟶ member satisfaction	0.001	0.048	0.001	0.048
SCC ⟶ organizational change ability ⟶ member satisfaction	0.004	0.036	0.004	0.036
CSC ⟶ environmental perception ⟶ economic benefits	0.085	0.231	0.085	0.224
CSC ⟶ organizational change ability ⟶ economic benefits	0.066	0.104	0.066	0.104
CSC ⟶ environmental perception ⟶ member satisfaction	0.109	0.381	0.104	0.369
CSC ⟶ organizational change ability ⟶ member satisfaction	0.045	0.231	0.045	0.247

## Data Availability

The data used to support the findings of this study are included within the article.
